The article "Prevalence of SARS-CoV-2 Antibodies in Laboratory Healthcare Workers at Assiut University Hospital, Egypt" was published in 2022. Journal: J Environ Public Health.

# Prevalence of SARS-CoV-2 Antibodies in Laboratory Healthcare Workers at Assiut University Hospital, Egypt

**DOI:** 10.1155/2022/7833623

**Published:** 2022-05-06

**Authors:** Azza M. Ezz Eldin, Dalia Tarik Kamal, Samar Salah Eldin, Mariam R. Elkhayat, Alaa M. Attia, Zeinab Ahmed Abd Elhameed

**Affiliations:** ^1^Clinical Pathology, Head of the Department, Assiut University Hospitals, Assiut, Egypt; ^2^Clinical Pathology, Assiut University Hospitals, Assiut, Egypt; ^3^Clinical Pathology Department, Assiut University Hospitals, Assiut, Egypt; ^4^Occupational & Environmental Medicine Department, Faculty of Medicine, Assiut University Hospitals, Assiut, Egypt; ^5^Anesthesia, Assiut University Hospitals, Assiut, Egypt

## Abstract

**Background:**

COVID-19 is an illness caused by a novel coronavirus known as severe acute respiratory syndrome coronavirus 2 (SARS-CoV-2). Laboratory healthcare workers (LHCWs) are at highest risk for COVID-19 infection due to direct exposure to COVID-19 patients and/or infected samples.

**Objectives:**

Our primary objective in this study was to evaluate SARS-CoV-2 Ab testing as a screening tool for detecting COVID-19 infection among asymptomatic LHCWs. Our secondary aims were to establish the relationship between exposure to COVID-19 infection and subsequent asymptomatic disease and working in different areas of the laboratory.

**Method:**

The detection of SARS-CoV-2 antibodies was done by different methods (rapid testing, electrochemiluminescence, and chemiluminescent microparticle immunoassay). The study included 199 asymptomatic LHCWs at Assiut University Hospital, Egypt, from different laboratory areas including molecular biology, microbiology, parasitology, and outpatient clinic laboratories in addition to LHCWs involved in automation, phlebotomy, rotating physicians, and those working in the sample receiving area.

**Results:**

The incidence of SARS-CoV-2 antibodies by rapid testing and immunoassay among asymptomatic LHCWs was 29.6% and 24.4%. Laboratory phlebotomists (55.6%) were most likely to be exposed to positive patients and samples, followed by those working in the sample receiving area (32%), LHCWs in the automation area (29.6%), rotating doctors (28.6%), and LHCWs in the diagnostic molecular biology laboratory (15.4%). The sensitivities of the rapid test and SARS-CoV-2 total antibody were 94.1% and 92%, whereas the specificities were 92.6% and 91%.

**Conclusion:**

Rapid serological testing is an effective screening method for the detection of SARS-CoV-2 infection among asymptomatic LHCWs and the identification of the groups of workers who have a significantly higher seroprevalence than the rest of the laboratory population.

The article "Prevalence of SARS-CoV-2 Antibodies in Laboratory Healthcare Workers at Assiut University Hospital, Egypt" was published in 2022. Journal: J Environ Public Health.

## 1. Introduction

COVID-19 is defined as an illness caused by a novel coronavirus now called severe acute respiratory syndrome coronavirus 2 (SARS-CoV-2), which was first identified as an outbreak of respiratory illness cases in Wuhan City, China, in December 2019 [1]. Lately, the novel SARS-CoV-2 has aggressively spread throughout the world, causing the COVID-19 pandemic which was declared as a public health emergency of international concern by the WHO [2]. SARS-CoV-2 is an enveloped single-stranded RNA virus, which is 29,881 bp. in length and encodes 9860 amino acids. The presence of SARS-CoV-2-specific antibodies strongly correlate with the molecular structure of the virus [3]. Changes in titer of both the IgM and IgG antibodies throughout the disease is sparse; however, the quantitative detection of antibodies has significant potential for evaluating the severity and prognosis of COVID-19 [4].

Healthcare workers are critical to the ongoing response to the SARS-CoV-2 pandemic. During their work, they are exposed to hazards that place them at risk of infection [5]. Laboratory health care workers (LHCWS) are exposed to hazards that place them at higher risk of infection, during sample collection or testing procedures in the lab. Previous studies have shown infection rates of up to 14% and 7.1% in symptomatic and asymptomatic healthcare workers, respectively, suggesting an occupational risk [6]. The detection of SARS-CoV-2 antibodies among healthcare workers is important since SARS-CoV-2 polymerase chain reaction (PCR) tests can only detect active infections. It is currently estimated that 25% of the cases are asymptomatic [7]. Serological tests, in theory, can provide a more accurate estimate of the rate of SARS-CoV-2 exposure amongst LHCWs than PCR. Also, it can help in conducting seroprevalence studies for community screening, epidemiological studies, and screening convalescent plasma collected from individuals who have recovered from COVID-19 [7].

The Centers for Disease Control and Prevention (CDC) and Occupational Health and Safety Administration (OSHA) have recommended using a combination of standard precautions, contact precautions, airborne precautions, and eye protection (e.g., goggles or face shields) to protect laboratory workers from exposure to the virus, especially those handling clinical specimens from patients with suspected or confirmed COVID-19 or samples of SARS-CoV-2 collected during research studies [8].

In this study, we evaluate the role of SARS-CoV-2 Ab testing as a screening method for detecting SARS-CoV-2 infections among LHCWs. We also determine the relationship between SARS-CoV-2 infection and various laboratory categories/areas.

The article "Prevalence of SARS-CoV-2 Antibodies in Laboratory Healthcare Workers at Assiut University Hospital, Egypt" was published in 2022. Journal: J Environ Public Health.

## 2. Methods

A cross-sectional study was aimed at all active laboratory healthcare workers (LHCWs) during the COVID-19 outbreak from April 2020 to June 2020 (first wave) at Assiut University Hospital labs (Egypt). We recruited a total of 199 asymptomatic LHCWs from different laboratory areas including molecular biology, microbiology, parasitology, and outpatient laboratories in addition to LHCWs working in automation, phlebotomy, rotating physicians, and those working in the sample receiving area. Symptomatic or suspected COVID-19 LHCWs and lab workers who refuse to share were excluded.

Before starting testing, we sought ethics approval from the Ethics Committee of the Assiut University Faculty of Medicine (no. 17101255) and registered as a clinical trial under ClinicalTrials.gov ID: NCT04445415. Individual written consent was also taken from every respondent, after discussing aims of research and confirmed that all samples will be coded for confidentiality and results will be in person informed by researcher, all of whom were told that they were free to decline to answer any question they opted not to answer or take samples.

Researchers convened and ran intervention design, specific admin room in Assiut university hospital labs was dedicated for sample collection and filling questionnaire by trained personal under supervision of researchers, and this was announced for all LHCWs. All samples were coded for conventionality, and participants were informed with their results personally by researcher. Time needed for each LHCWs was nearly 20 min for filling the questionnaire and sample procedure discussed in Figure 1.

Interviewed questionnaire included questions about three parts: the first part was sociodemographic characteristics such as age, gender, and residence; the second part on occupational exposure history as job title, working area, PPE using, and previous history of dealing with COVID-19 specimen; last part, asking about risk factors of COVID-19 infections warned by WHO as previous contact with infected family member and using public or private transportation.

The primary outcomes were percentages of infected COVID-19 LHCWs in each area in Assiut University Hospital different labs and find the association between variable exposures with being COVID-19 infection.

### 2.1. Sample Collection

Whole blood samples (5 ml) were collected using venipuncture. 3 ml was added to a gel and clot activator tube for separating sera. The remaining 2 ml was placed into an EDTA tube for complete blood cell count including WBCs and lymphocytes. Oropharyngeal and nasopharyngeal swabs were collected for SARS-CoV-2 diagnosis and viral clearance was evaluated by real-time PCR. A questionnaire was provided to all participants asking about their possible exposure to SARS-CoV-2 infection. Complete blood count (CBC) was performed using an Advia 2120 hematology analyzer (Siemens Healthcare).

The article "Prevalence of SARS-CoV-2 Antibodies in Laboratory Healthcare Workers at Assiut University Hospital, Egypt" was published in 2022. Journal: J Environ Public Health.

### 2.2. COVID-19-Specific Antibody

The detection of SARS-CoV-2 antibodies was performed by three different methods (rapid testing, electrochemiluminescence, and chemiluminescent microparticle immunoassay immunoassay). The detection of SARS-CoV-2 IgM and IgG antibodies by rapid testing was performed using a kit obtained from Artron (One Step Rapid Diagnostic Test, Lot No. SR200302 London, United Kingdom) based on an immunochromatographic assay. The test card contained a colloidal gold-labeled recombinant novel coronavirus antigen and quality control antibody gold markers, two detection lines (IgG and IgM lines), and one quality control line on a nitrocellulose membrane. The lines were immobilized with a monoclonal anti-human IgM and IgG antibody for detecting novel coronavirus IgM and IgG, and the control line was immobilized with a quality control antibody.

A quantitative assay for SARS-CoV-2 total antibody was performed using a kit obtained from Roche Diagnostics (Elecsys Anti-SARS-CoV-2 kit, lot no. 49546401, Germany) based on an electrochemiluminescence immunoassay “ECLIA” using a COBAS E 411 immunoassay analyzer. The detection of SARS-CoV-2 IgG antibody was performed using the SARS-CoV-2 IgG kit (lot no. 18099FN00, Abbott diagnostics) based on chemiluminescent microparticle immunoassay (CMIA) technology using an ARCHITECT i1000SR analyzer. This assay is an automated, two-step immunoassay for the qualitative detection of IgG antibodies against SARS-CoV-2 in human serum and plasma using SARS-CoV-2 antigen-coated paramagnetic microparticles.

To detect positive SARS-CoV-2 IgM in LHCWs, an RT-PCR assay was performed for the detection of SARS-CoV-2 RNA. For RNA extraction, nasopharyngeal and oropharyngeal swabs were collected according to CDC guidelines that involved inserting a swab into the nostril, parallel to the palate, leaving the swab in place for several seconds to absorb secretions, and slowly rotating and removing the swab. After sample collection, the swabs were placed into 2 mL of sterile viral transport medium (VTM; various manufacturers). The samples were transported to the Immunology and Molecular Virology Laboratory within 12 h after collection and tested immediately. RNA extraction from nasopharyngeal and oropharyngeal samples was done using the Qiagen RNA extraction kit (lot no. HB-0354-0007) and a QIAcube fully automated nucleic acid purification system. The detection of SARS-CoV-2 RNA was performed using the Genesig® Real-Time PCR Coronavirus SARS-CoV-2 (CE IVD) real-time PCR kit (Issue 3.0) obtained from Primerdesign TM Ltd. (United Kingdom) using an Applied Biosystems® 7500 Real-Time PCR instrument.

The article "Prevalence of SARS-CoV-2 Antibodies in Laboratory Healthcare Workers at Assiut University Hospital, Egypt" was published in 2022. Journal: J Environ Public Health.

### 2.3. Statistical Analysis

Data were analyzed by IBM SPSS V22 software. Descriptive statistics were calculated as frequency and percentage. A Chi-square test was also used for comparing different predictors of the SARS-CoV-2 test results. Tests were considered significant if *p* values were less than 0.05. Sensitivity, specificity, and positive and negative predictive values (PPV/NPV) were performed across the different lab tests for significance.

## 3. Results

Here, we present data from 199 asymptomatic laboratory HCWs. The rapid test for SARS-CoV-2 IgG and IgM was done on all individuals (Figure 2). The results indicated that 140 (70.4%) were negative and 59 (29.6%) were positive (34 (57.6%) were SARS-CoV-2 IgG Ab positive, 21 (35.6%) were SARS-CoV-2 IgM Ab positive, and 4 (6.8%) were positive for both). PCR was done for individuals who expressed SARS-CoV-2 IgM, 11 were positive and 10 were negative for SARS-CoV-2 RNA.  Table 1 presents the relative percentages of rapid test and PCR positive results in relation to gender, residence, work area, contact with COVID-19 specimens, and family history of COVID-19.

Total Ab for SARS-CoV-2 was determined for all participants in the study (Figure 3), 148 (74.4%) were negative, and 51 (25.6%) were positive. SARS-CoV-2 IgG Ab was tested in participants who had total SARS-CoV-2 Ab, and 39 were positive, whereas 12 were negative.  Table 2 presents the relative percentages of total SARS-CoV-2 Ab and IgG Ab relative to gender, residence, work area, working with COVID-19 specimens, and family history of COVID-19.

Statistical tests revealed no statistically significant differences among these categories of risk. The sensitivity, specificity, and positive and negative predictive values for the rapid test, WBCs, and total Ab are presented in Table 3.

The results of the rapid test (Table 1) indicate that approximately one-third of males and females were COVID-19 positive. With respect to working environment, the phlebotomy area recorded the highest infection rate (55.5%), followed by the microbiology lab, sample receiving area, and automation area. These areas recorded nearly one-third of the positive LHCWs tests, followed by outpatient clinic LHCWs in which nearly a quarter were positive. The lowest percentage of infections was observed in the PCR and parasitology labs. One-third of the doctors tested positive. Among the PCR results, males exhibited a statistically significant higher infection rate than females (69.2% vs. 25%), although other characteristics were not significant. 62.5% of LHCWs who had a history of exposure to SARS-CoV-2 specimens were positive PCR versus 20% that did not deal with such specimens.

The article "Prevalence of SARS-CoV-2 Antibodies in Laboratory Healthcare Workers at Assiut University Hospital, Egypt" was published in 2022. Journal: J Environ Public Health.

Table 2 lists the effect of sociodemographic features, transportation, and occupational exposure on SARS-CoV-2 total and IgG antibody results. None of the variables showed a statistically significant difference; however, 100% of LHCWs associated with the PCR lab, parasitology lab, and phlebotomy tested positive for SARS-CoV-2 IgG antibody, and 83% of rotating physicians tested positive for the SARS-CoV-2 IgG antibody.

Table 4 illustrates the relationship between the results of the SARS-CoV-2 rapid and total antibody testing. The results indicate that 97.9% of the LHCWs who tested negative in the rapid test exhibited a negative total antibody test, whereas only 81.4% of the LHCWs who tested positive in the rapid test had a positive total antibody test.

Table 3 lists the sensitivity, specificity, positive predictive value, and negative predictive value for WBCs, the SARS-CoV-2 rapid test, and total antibody results. The rapid test showed the highest level of sensitivity and specificity (94% and 93%). In contrast, the WBC test was associated with the lowest sensitivity (13.6%).

## 4. Discussion

In this study, the incidence of SARS-CoV-2 antibodies identified by rapid testing and immunoassay among asymptomatic LHCWs was 29.6% and 24.4%, respectively. This is consistent with the results of Shields et al. who demonstrated that the positivity of serological SARS-CoV-2 antibody testing in HCWs is between 23.8% and 26.0% [7]. Other studies also revealed higher seroprevalence or rates of asymptomatic infection in healthcare workers compared with the general population [9, 10]. Collectively, these studies suggest a marked occupational risk of exposure to SARS-CoV-2 associated with laboratory healthcare work during the COVID-19 pandemic.

Our study also revealed that the group most at risk was phlebotomy (55.6%), followed by those working in the sample receiving area (32%), automation area (29.6%), rotating physicians (28.6%), and the diagnostic molecular biology laboratory (15.4%). The highest infection rate was observed in phlebotomy and workers in the sample receiving area due to direct exposure to COVID-19 patients or infected samples. A lower seroprevalence was observed in the diagnostic molecular biology laboratory. This strongly supports the conclusion that a varying risk of SARS-CoV-2 exposure exists within the hospital environment. The reasons underlying this are likely to be multifactorial. Assiut University guidelines established designated high-risk environments and the use of enhanced personal protective equipment (PPE) including mask N95, face shields, shoe covers, and gowns in addition to continuous training. In contrast, only fluid-resistant surgical masks were recommended in other areas. The contribution of enhanced PPE in protecting staff from infection with SARS-CoV-2 should be studied further including the availability of training, space, and supervision for effectively using PPE [11].

The article "Prevalence of SARS-CoV-2 Antibodies in Laboratory Healthcare Workers at Assiut University Hospital, Egypt" was published in 2022. Journal: J Environ Public Health.

The percent of PCR positive results in all the study groups was 11 out of 199 (5.5%). A screening study of asymptomatic healthcare workers revealed that 3% were PCR positive using pharyngeal swab specimens [12]. Similar findings were observed in a Dutch study of 1,353 healthcare workers wherein 86 (6%) tested positive for SARS-CoV-2 using nasal swab specimens [13]. The most infected groups were workers in the outpatient clinic (3), automation area (3), PCR lab (2), and sample receiving area (2). All these individuals were working directly with COVID-19 samples (Table 1). These results emphasize the importance of using PPE in the lab, especially when working with COVID-19 samples or other highly virulent respiratory pathogens.

The sensitivity and specificity of SARS-CoV-2 antibody rapid testing was 94.1% and 92.6%, respectively. This is in agreement with Silva et al. who reported that the sensitivity and specificity of the rapid test was 86.43% and 99.57%, respectively [14]. Li et al. reported that the sensitivity was 88.66% and the specificity was 90.63% [15]; however, there were still false-positive and false‐negative results. False-negative results may result from low antibody concentrations in which Ab levels are below the detection limit of the rapid test, causing the results to be negative. Also, the difference in individual immune response and antibody production could be a reason for the false‐negative results. Abs may not yet be generated during the early stages of infection, and SARS-CoV-2 IgM antibodies may decrease and disappear after 2 weeks. Therefore, the optimum time of testing is very important, especially in asymptomatic individuals [15]. False positives can result from cross‐reactivity with preexisting antibodies from previous infections, such as other coronaviruses that cause common cold [16].

Rapid tests for COVID-19 are attractive for large seroprevalence studies and can be used as point-of-care tests [17]. Diao et al. reported that a fluorescence immunochromatographic assay is an accurate, rapid, early, and simple method for detecting the nucleocapsid protein of SARS-CoV-2 and in the diagnosis of COVID-19. Our results indicate that the sensitivities of the rapid test, total SARS-CoV-2 Ab, and IgG Ab were 94.1%, 92%, and 73.7%, respectively, whereas the specificities were 92.6%, 91%, and 93.2%, respectively. The combined SARS-CoV-2 IgG/IgM test displayed better sensitivity than measuring either antibody type alone [17]. A recent study revealed a high sensitivity and specificity of the SARS‐CoV‐2 neutralizing antibodies [18]. A meta-analysis showed that all serological tests have high specificity, especially the ELISA and rapid test, which can reach levels higher than 99%. ELISA- and CLIA-based methods performed better in terms of sensitivity (90%–96%) followed by the rapid test with sensitivities ranging from 80% to 89% [17]. As such, the total Ab test may be replaced with the rapid test for the screening of asymptomatic HCWs to help prevent transmission [19]. Finally, WBCs exhibited a very low sensitivity (13.6%) with high specificity (91.4%), indicating that it is not worth considering as a screening test for asymptomatic individuals.

The article "Prevalence of SARS-CoV-2 Antibodies in Laboratory Healthcare Workers at Assiut University Hospital, Egypt" was published in 2022. Journal: J Environ Public Health.

In conclusion, we found that rapid serological tests for SARS-CoV-2 antibodies are essential in determining the SARS-CoV-2 antibody status among asymptomatic laboratory healthcare workers. Moreover, they can identify groups of workers who have significantly different seroprevalence, suggesting a varying occupational risk.

### 4.1. Recommendations

Further studies are required to confirm and fully interpret our findings and to propose an optimal utilization of serological tests in clinical settings. The contribution of enhanced PPE in protecting staff from infection should be studied further including the availability of training, space, and supervision for effectively using PPE among HCWS.

## Figures and Tables

**Figure 1:** Timeline and steps of research.

**Figure 2:** SARS-CoV-2 antibodies and RNA in asymptomatic laboratory HCWs.

**Figure 3:** SARS-CoV-2 total and IgG antibody results in asymptomatic LHCWs.

**Table 1:** Effect of sociodemographic, transportation, and occupational exposure history on SARS-CoV-2 antibodies and RNA results.

Characteristics	Total *N* (%) (199)	Rapid test (199)					PCR (21)	
		Negative (140)	Positive (59)	IgG (34)	IgM (21)	Combined (4)	Negative (10)	Positive (11)
Gender								
Male	74 (37.2%)	50 (67.6%)	24 (32.4%)	14	8	2	6 (30.8%)	2 (69.2%)^*∗*^
Female	125 (62.8%)	90 (72%)	35 (28%)	20	13	2	4 (75.0%)	9 (25.0%)
Age groups								
22–32 Ys	84 (42.2%)	60 (71.4%)	24 (28.6%)	15	9	0	2 (40.0%)	3 (60.0%)
33–43 Ys	68 (34.1%)	46 (67.6%)	22 (32.4%)	15	5	2	6 (66.7%)	3 (33.3%)
44–59 Ys	47 (23.7%)	34 (72.3%)	13 (27.7%)	4	7	2	2 (28.6%)	5 (71.4%)
Residence								
Urban	128 (64.3%)	85 (66.4%)	43 (33.6%)	25	14	4	7 (50.0%)	7 (50.0%)
Rural	71 (35.7%)	55 (77.5%)	16 (22.5%)	9	7	0	3 (42.9%)	4 (57.1%)
Work area								
Doctors	28 (14.1%)	20 (71.4%)	8 (28.6%)	5	3	0	2 (66.7%)	1 (33.3%)
PCR lab	13 (6.5%)	11 (84.6%)	2 (15.4%)	0	2	0	0 (0.0%)	2 (100%)
Microbiology lab	18 (9%)	12 (66.7%)	6 (33.3%)	4	1	1	1 (100%)	0
Parasitology lab	10 (5%)	9 (90%)	1 (10%)	1	0	0	—	—
Phlebotomy	9 (4.5%)	4 (44.4%)	5 (55.6%)	3	1	1	1 (100%)	0 (0.0%)
Outpatient clinic	19 (9.5%)	14 (73.7%)	5 (26.3%)	0	5	0	2 (40.0%)	3 (60.0%)
Sample receiving area	50 (25.1%)	34 (68%)	16 (32%)	11	4	1	2 (50.0%)	2 (50.0%)
Automation area	52 (26.1%)	36 (70.4%)	16 (29.6%)	10	5	1	2 (40.0%)	3 (60.0%)
Deal with COVID-19 specimen								
Yes	120 (60.3%)	82 (68.3%)	38 (31.7%)	20	16	2	6 (37.5%)	10 (62.5%)
No	79 (39.7%)	58 (73.4%)	21 (26.6%)	14	5	2	4 (80.0%)	1 (20%)
Transportation								
Private	61 (30.7%)	43 (70.4%)	18 (29.6%)	13	5	0	4 (80.0%)	1 (20.0%)
Public	138 (69.3%)	99 (71.7%)	39 (28.3%)	20	16	3	6 (37.5%)	10 (62.5%)
Had family COVID-19 contact								
Yes	69 (34.6%)	45 (65.2%)	24 (34.8%)	13	10	1	4 (40%)	6 (60%)
No	130 (65.4%)	95 (73.1%)	35 (26.9%)	21	11	3	6 (54.5%)	5 (45.5%)

All were statistically insignificant (*p* > 0.05) except ^*∗*^significant *p* (<0.05).

The article "Prevalence of SARS-CoV-2 Antibodies in Laboratory Healthcare Workers at Assiut University Hospital, Egypt" was published in 2022. Journal: J Environ Public Health.

**Table 2:** Effect of sociodemographic, transportation, and occupational exposure history on SARS-CoV-2 total and IgG antibodies results.

Characteristics	Total *N* (%) (199)	Total Ab (199)		IgG Ab (51)	
		Negative (148)	Positive (51)	Negative (12)	Positive (39)
Gender					
Male	74 (62.8%)	54 (73%)	20 (27%)	3 (29.0%)	17 (71.0%)
Female	125 (37.2%)	94 (75.2%)	31 (24.8%)	9 (15.0%)	22 (85.0%)
Age groups					
22–32 Ys	84 (42.2%)	60 (71.4%)	24 (28.6%)	7 (41.2%)	10 (58.8%)
33–43 Ys	68 (34.1%)	53 (77.9%)	15 (22.1%)	3 (14.3%)	18 (85.7%)
44–59 Ys	47 (23.7%)	35 (74.5%)	12 (25.5%)	2 (15.4%)	11 (84.6%)
Residence					
Urban	128 (64.3%)	90 (70.3%)	38 (29.7%)	10 (26.3%)	28 (73.7%)
Rural	71 (35.7%)	58 (81.7%)	13 (18.1%)	2 (15.4%)	11 (84.6%)
Job area					
Doctors	28 (14.1%)	22 (78.6%)	6 (21.4%)	1 (16.7%)	5 (83.3%)
PCR lab	13 (6.5%)	12 (92.3%)	1 (7.7%)	0 (0.0%)	1 (100%)
Microbiology lab	18 (9%)	13 (72.2%)	5 (27.8%)	3 (60.0%)	2 (40.0%)
Parasitology lab	10 (5%)	9 (90%)	1 (10%)	0 (0.0%)	1 (100%)
Phlebotomy	9 (4.5%)	5 (55.5%)	4 (44.5%)	0 (0.0%)	4 (100%)
Outpatient clinic	19 (9.5%)	15 (79%)	4 (21%)	2 (50.0%)	2 (50.0%)
Sample receiving area	50 (25.1%)	36 (72%)	14 (28%)	3 (21.4%)	11 (78.6%)
Automation area	52 (26.1%)	36 (69.2%)	16 (30.8%)	3 (18.8%)	13 (81.2%)
Deal with COVID-19 specimen					
Yes	120 (60.3%)	89 (74.2%)	31 (25.8%)	6 (29.4%)	25 (80.6%)
No	79 (39.7%)	59 (74.7%)	20 (25.3%)	6 (30.0%)	14 (70.0%)
Transportation					
Private	61 (30.7%)	48 (78.6%)	13 (21.4%)	2 (8.3%)	11 (91.7%)
Public	138 (69.3%)	100 (72.5%)	38 (27.5%)	10 (27.0%)	28 (73.0%)
Had family COVID-19 contact					
Yes	69 (34.6%)	50 (72.5%)	19 (27.5%)	3 (15.8%)	16 (84.2%)
No	130 (65.4%)	98 (75.4%)	32 (24.6%)	9 (28.1%)	23 (71.9%)

The article "Prevalence of SARS-CoV-2 Antibodies in Laboratory Healthcare Workers at Assiut University Hospital, Egypt" was published in 2022. Journal: J Environ Public Health.

**Table 3:** Sensitivity, specificity, positive predictive value, and negative predictive value for WBCS, SARS-CoV-2 rapid and total antibody testing.

	Sensitivity (%)	Specificity (%)	PPV (%)	NPV (%)
WBCs	13.6	91.4	40	71.5
Rapid test	94.1	92.6	81.4	97.8
Total Ab	92	91	83	96.6

**Table 4:** Relation between SARS-CoV-2 rapid and total antibody testing.

	Total antibody test (199)	
	Negative (148)	Positive (51)
Rapid test, *N* = 199		
(i) Negative (140)	137 (97.9%)	3 (2.1%)
(ii) Positive (59)	11 (18.6%)	48 (81.4%)

## Data Availability

Data are available upon request.
